RETRACTED

# Dapagliflozin Inhibits Ventricular Remodeling in Heart Failure Rats by Activating Autophagy through AMPK/mTOR Pathway

**DOI:** 10.1155/2022/6260202

**Published:** 2022-09-23

**Authors:** Honghong Ma, Yanmei Ma

**Affiliations:** ^1^Department of Cardiovascular Medicine, The First Hospital of Yulin, Yulin, 719000 Shaanxi, China; ^2^Department of Pathology, The First Hospital of Yulin, Yulin, 719000 Shaanxi, China

## Abstract

**Objective:**

Heart failure (HF) is the end stage of heart disease caused by various factors which mainly involves ventricular remodeling (VR). In HF patients with reduced ejection fraction, dapagliflozin (DAPA) reduced the risk of worsening HF or cardiovascular death. Thus, we attempted to clarify the specific role of DAPA underlying HF progression.

**Methods:**

The HF rat model was established to mimic characteristics of HF in vivo. HE staining assessed histopathological changes in left ventricular myocardial tissue of rats in each group. ELISA measured plasma ANP and BNP levels of rats in each group. M-mode echocardiography detected cardiac function of rats in each group. TUNEL staining detected apoptosis of infarct margin cells in myocardial tissue of rats in each group. Western blot detected levels of apoptosis-related proteins, autophagy-related proteins, and AMPK/mTOR-related proteins in myocardial tissue of rats in each group. Immunohistochemical staining detected caspase-3 or LC3B level in myocardial tissue of rats in each group. The HF cellular model was established to mimic characteristics of HF in vitro. Flow cytometry detected H9C2 cell apoptosis under different conditions. Western blot detected levels of apoptosis-related proteins, autophagy-related proteins, and AMPK/mTOR-related proteins in H9C2 cells under different conditions. Immunofluorescence detected caspase-3 or LC3B level in H9C2 cells under different conditions.

**Results:**

DAPA attenuated left VR and improved cardiac function in HF rats. DAPA attenuated cardiomyocyte apoptosis in HF rats. DAPA facilitated cardiomyocyte autophagy in HF rats via the AMPK/mTOR pathway. DAPA repressed hypoxia-induced H9C2 cell apoptosis by facilitating autophagy. DAPA repressed hypoxia-induced H9C2 cell apoptosis via the AMPK/mTOR pathway.

**Conclusion:**

DAPA suppresses ventricular remodeling in HF through activating autophagy via AMPK/mTOR pathway, which provides a potential novel insight for seeking therapeutic plans of HF.

## 1. Introduction

Heart failure (HF) is the end stage of heart disease caused by various factors [1], and its pathological mechanism is complex. Currently, it mainly involves ventricular remodeling (VR) and excessive activation of the neuroendocrine system [2, 3]. Though the therapy of HF has made great advancement in recent years, the mortality and readmission rates of patients are still quite high [4]. It is necessary to figure out new intervention targets, pathways, and treatment means for HF.

RETRACTED

VR is a compensatory mechanism in HF, but simultaneously, it changes the function of myocardium and accelerates the process of HF. Additionally, myocardial remodeling is the result of the combination of myocardial apoptosis, myocardial hypertrophy, and myocardial fibrosis [5]. There is accumulation of misfolded proteins and damaged organelles in hypertrophic cardiomyocytes [6], and autophagy can specifically remove misfolded proteins and damaged organelles, reducing their damage to cardiomyocytes [7]. The autophagy agonist, rapamycin, improved myocardial fibrosis and cardiac function in HF rats; when chloroquine was given to suppress autophagy, myocardial fibrosis in rats was aggravated and cardiac function deteriorated [8]. Through researching the hearts of dilated cardiomyopathy patients, Andres et al. demonstrated that autophagosome formation had positive association with better prognosis of chronic HF [9], confirming the protective role of autophagy underlying HF. It can be seen that autophagy activation may be one of the reasons for retarding HF, and the mechanism may be that cardiomyocyte autophagy can delay VR and elevate cardiac function. Thus, elevating autophagy level in myocardial tissue may be a vital link in the prevention and therapy of HF.

AMP-activated protein kinase (AMPK) is a serine-threonine kinase that plays an important role in maintaining energy homeostasis during cellular stress [10]. Activation of AMPK can trigger autophagy by inhibiting rapamycin (mTOR) through mammalian target proteins [11]. AMPK/mTOR pathway plays a crucial role in HF [12].

Sodium-glucose cotransporter 2 (SGLT2) inhibitor (SGLT2i) is a novel hypoglycemic drug facilitating excretion of glucose from urine by suppressing SGLT2, which mediates glucose reabsorption in renal proximal tubule [13]. Besides its hypoglycemic impact, SGLT2i, can also exert a cardioprotective role [14]. In patients with HF and reduction of ejection fraction, dapagliflozin (DAPA), a type of SGLT2i, reduced the risk of worsening HF or cardiovascular death [15]. Furthermore, the *2021 ESC Guidelines for the diagnosis and treatment of acute and chronic heart failure* included DAPA as one of the category I recommendations for therapy of HF patients with reduced ejection fraction to attenuate the risk of hospitalization and death in HF patients [16]. Currently, it has been revealed that DAPA restores autophagy through the AMPK-mTOR pathway, thereby alleviating hepatic steatosis [17], whereas there is no report that DAPA facilitates autophagy in HF. Thus, we wondered whether DAPA suppressed VR in HF rats through activating autophagy via the AMPK/mTOR pathway.

RETRACTED

Herein, we attempted to figure out DAPA role underlying autophagy in HF progression and clarify the potential downstream pathways, which may provide a novel insight for targeted therapy of HF.

## 2. Materials and Methods

### 2.1. Animal Models

A total of 30 Sprague-Dawley (SD) male rats (220 ± 10 g) were provided by Beijing Vital River Laboratory Animal Technology Co., Ltd. The rats were divided into three groups (*n* = 10 rats/group): control, model, and DAPA. All rats received intraperitoneal anesthetization with 1% pentobarbital sodium at 50 mg/kg. The rats in the control group received sham surgery, and the other two groups had the anterior descending coronary artery (LAD). The left LAD of the rats was ligated to establish the HF models as described before [18]. Briefly, left thoracotomy was performed between the third and fourth intercostal space with the heart exposed. The LAD was ligated 1–1.5 mm proximal to the main diagonal branch and sutured aseptically. The box was closed, and the rats were placed on thermal blankets. After 24 h, the DAPA group received DAPA by gavage at 5 mg/kg/day for four consecutive weeks, and the other two groups received the same amount of normal saline. During whole procedure, none of rats died after surgery or during surgery. The assays were performed according to the Guide for the Institutional Animal Care and Use Committee. The Animal Care Committee of our hospital approved this research.

### 2.2. Histological Detection

After hearts were harvested, left ventricular (LV) were separated and weighed. The heart weight (HW) to tibial length (TL) (HW/TL, g/cm) and LV weight (LVW) to TL (LVW/TL, g/cm) ratios received calculation. The myocardial tissues got fixation with 4% paraformaldehyde for 72 h, embedding in paraffin and cutting into 5 mm slices. The paraffin section received staining with hematoxylin-eosin (HE). The changes were observed under an optical microscope (×400; Leica Microsystems).

### 2.3. Enzyme-Linked Immunosorbent Assay (ELISA)

Circulating vasoactive peptide contents were measured via ELISA kits under manufacturer's guidance. The serum levels of atrial natriuretic peptide (ANP; Uscnk, Wuhan, China) and brain natriuretic peptide (BNP) were examined.

### 2.4. Echocardiography

The rats received intraperitoneal anesthetization with 1% pentobarbital sodium at 50 mg/kg. The LV cardiac function of rats was recorded by echocardiography in 2D M-mode (Visual Sonics, Canada). LV internal diameter at end-diastole (LVIDd), LV internal diameter at end-systole (LVIDs), ejection fraction (EF), and fractional shortening (FS) were measured for at least three consecutive cardiac cycles: EF = [(LVEDv–LVESv)/LVEDv] × 100% and FS = [(LVEDd–LVESd)/LVEDd] × 100%.

RETRACTED

### 2.5. TUNEL

Tissue sections (4 *μ*m thickness) were dewaxed with xylene, rehydrated with ethanol, and incubated with proteinase K for 20 min. The apoptosis was assessed by TUNEL assay under manufacturer's guidance (Roche, Germany). Nuclear staining with DAPI was also performed to quantify cell numbers. Images were chosen in a random manner and then analyzed.

### 2.6. Cell Lines and Cell Culture

H9C2 cells provided by Procell (Wuhan, China) were cultured in DMEM containing 1% antibiotics (100 U/ml penicillin and 100 *μ*g/ml streptomycin) and 10% fetal bovine serum at 37°C with 5% CO_2_. To induce the HF in vitro model, H9C2 cells were seeded into 96-well plates. After 24 h, cell density reached about 80%. H_2_O_2_ was given (100 *μ*mol/L) for culture for 4 h, and then original medium was discarded. Each well received treatment with DMEM (Corning, USA). H9C2 cells were divided into different groups: control, H/R, H/R + DAPA, and DAPA+compound C (Comp C). Comp C (20 *μ*M, Sigma-Aldrich, USA), an inhibitor of AMPK, was set as positive drug.

### 2.7. Western Blot

Total protein got extraction from rat myocardial tissues at infarcted margin area and the cultured H92C cells through RIPA lysis buffer. Protein quantification was conducted through a BCA kit. The protein concentration was determined by the BCA method. The 5× SDS gel electrophoresis buffer was added and denatured at 100°C for 10 min. After completely separated by electrophoresis, the protein was transferred to the PVDF membrane by the semidry method. After blocked by 5% skimmed milk powder at room temperature for 2 h, the specific primary antibodies (cleaved caspase-3 (ab32042, 1/500), cleaved caspase-7 (ab256469, 1/1000), LC3B-I/II (ab63817, 1 *μ*g/ml), beclin-1 (ab207612, 1/2000), p62 (ab207305, 1/1000), p-AMPK (ab92701, 1/1000), AMPK (ab32047, 1/1000), p-mTOR (ab109268, 1/1000), mTOR (ab134903, 1/10000), and *β*-actin (ab115777, 1/200); Abcam, Shanghai, China) were added and incubated overnight at 4°C. Then, the secondary antibodies (ab205718, 1/2000) were added, incubated for another 2 h, and washed with TBS. Absorbance analysis was performed after color development to calculate relative expression of each protein.

### 2.8. Immunochemistry (IHC)

Dewaxed and rehydrated mouse lung tumor slides received treatment of 3% hydrogen peroxide and 5% BSA. The slides received incubation with primary antibody anti-caspase-3 (ab32351, 1/25) or anti-LC3B (ab239416, 5 *μ*g/ml) overnight and received subsequent incubation with a secondary antibody for 30 min at room temperature. Sections were counterstained with hematoxylin and observed through microscopy.

RETRACTED

### 2.9. Flow Cytometry

The apoptosis was detected by combined Annexin V-FITC/PI double staining method (Thermo Fisher Scientific, USA). H9C2 cells were seeded into cell plates for culture. After washing with PBS 3 times, 5 *μ*l of Annexin V-FITC and 10 *μ*l of PI were added, respectively, mixed well, and reacted for 10 min at room temperature in the dark. FITC+ and PI− cells were defined as apoptotic cells. The apoptosis rate was measured on a flow cytometer.

### 2.10. Immunofluorescence

H9C2 cells were seeded into 6-well plates. After 24 h of incubation, cells received fixation with 4% paraformaldehyde for 20 min and then washed using PBS for three times. The 0.3% Triton X-100 broke cell membrane and 1% BSA buffer with 5% anti-goat serum blocked cells under room temperature for 1 h. FITC-labeled RNA probes applied were anti-caspase-3 (ab32351, 1/500) or anti-LC3B (ab239416, 0.1 *μ*g/ml). Olympus FluoView FV1000 confocal microscope was applied for images.

### 2.11. Statistical Analysis

SPSS 20.0 software processed data. The data were expressed as mean ± standard deviation (*m* ± *s*). The mean of samples between groups was compared using *t*-test and that of multiple groups through one-way analysis of variance followed by Tukey's post hoc test. All assays were conducted for three times. The difference was statistically significant upon *p* < 0.05.

## 3. Results

### 3.1. DAPA Attenuates Left VR and Improves Cardiac Function in HF Rats

Previously, in HF patients with reduced ejection fraction, DAPA reduced the risk of worsening HF or cardiovascular death [15]. Thus, we attempted to clarify the specific role of DAPA underlying HF progression. SD rats were divided into three groups: control, model and DAPA. The rats in the control group received sham surgery, and the other two groups had the LAD ligated at 1-1.5 mm from the left atrial appendage of rats. After 24 h, the DAPA group received DAPA by gavage at 5 mg/kg/day for four consecutive weeks, and the other two groups received the same amount of normal saline. HE staining clearly showed the pathological changes in myocardial tissue of rats. As a result, the left ventricular myocardial fibers were arranged neatly as well as tissue density, and cell morphology was regular in the control group; the left ventricular myocardial fibers were arranged loosely, and cell morphology were irregular in the model group, while DAPA treatment markedly reversed these pathological changes (Figure 1(a)). Moreover, the elevated diameter of cardiomyocytes were discovered in HF hearts, which showed depletion after DAPA stimulation (Figure 1(b)). Additionally, model rats presented elevation in HW, LVW, HW/TL, and LVW/TL relative to controls while DAPA rescued these changes (Figures 1(c)–1(f)). We also measured plasma ANP and BNP levels through ELISA. ANP and BNP levels presented elevation in the model group relative to the control group; DAPA treatment remarkably reduced abovementioned parameters to certain extent (Figures 1(g) and 1(h)). Then, we clarified DAPA impact on cardiac structure and function in model rats. M-mode echocardiography demonstrated the structural changes and systolic and diastolic dysfunction in model rats, as evidenced by increase in LVIDs and LVIDd and decrease in EF and FS, and these effects were countervailed by DAPA stimulation (Figures 1(i)–1(m)). Collectively, DAPA hinders left VR and benefits cardiac function in HF progression.

RETRACTED

### 3.2. DAPA Attenuates Cardiomyocyte Apoptosis in HF Rats

Apoptosis is a form of programmed cell death causing orderly and efficient removal of damaged cells [19]. To clarify DAPA influence on cardiomyocyte apoptosis in rats, TUNEL staining was conducted. The cardiomyocyte apoptosis rate in infarct margin of myocardial tissue from model rats presented elevation relative to controls, whereas DAPA treatment reversed this effect (Figure 2(a)). Moreover, western blotting further supported these results via measuring abundances of apoptosis-related proteins. We discovered that caspase-3/7 protein abundances in infarct margin of myocardial tissue showed upregulation in the model group relative to controls, while caspase-3/7 protein abundances in infarct margin of myocardial tissue showed downregulation in the DAPA group relative to the model group (Figure 2(b)). IHC results showed a similar trend of the caspase-3 expression to western blot results (Figure 2(c)). Collectively, DAPA suppresses cardiomyocyte apoptosis in vivo.

### 3.3. DAPA Facilitates Cardiomyocyte Autophagy in HF Rats via the AMPK/mTOR Pathway

Previously, DAPA ameliorated HG-triggered autophagy impairment in HK-2 cells [20]. DAPA restores autophagy through the AMPK-mTOR pathway, thereby alleviating hepatic steatosis [17]. Thus, we attempted to clarify whether DAPA activated autophagy pathway and the AMPK/mTOR signaling. LC3B is an adapter protein mediating vital protein-protein interactions in autophagy pathways [21]. Thus, we examined LC3B expression changes in myocardial tissue of rats using IHC. As a result, LC3B showed downregulation in myocardial tissue of model rats relative to controls and then got elevation under DAPA treatment (Figure 3(a)). Western blotting also demonstrated that LC3B-II/I and beclin-1 protein abundances presented depletion, whereas p62 showed upregulation in myocardial tissue of model rats relative to controls and then were rescued under DAPA treatment (Figure 3(b)), supporting the autophagy pathway activation under DAPA stimulation in vivo. Moreover, western blotting illustrated the downregulation of p-AMPK protein abundance and upregulation of p-mTOR protein abundance in myocardial tissue of model rats relative to controls and were reversed after DAPA treatment (Figure 3(c)). Collectively, DAPA exerts a promoting impact on cardiomyocyte autophagy in HF rats through the AMPK/mTOR pathway.

RETRACTED

### 3.4. DAPA Represses Hypoxia-Induced H9C2 Cell Apoptosis by Facilitating Autophagy

The abovementioned findings revealed the role of DAPA underlying VR and cardiac function in vivo. Thus, we aimed to clarify DAPA impact on cellular behaviors in vitro. A cellular model of HF was established to mimic HF characteristics in H9C2 cells under hypoxia. We assessed H9C2 cell apoptosis using flow cytometry. As a result, hypoxia triggered the elevation of H9C2 cell apoptosis and DAPA countervailed this influence (Figure 4(a)). Similarly, western blotting illustrated that caspase-3/7 protein abundances presented elevation in H9C2 cells under hypoxia and were rescued after DAPA stimulation (Figure 4(b)). IF staining showed a similar trend of the caspase-3 expression to western blotting results (Figure 4(c)). Furthermore, IF staining demonstrated that LC3B presented downregulation in hypoxia-treated H9C2 cells relative to controls and then got elevation under DAPA treatment (Figure 4(d)). Western blotting also illustrated that LC3B-II/I and beclin-1 protein abundances presented depletion, whereas p62 showed upregulation in H9C2 cells under hypoxia relative to controls, and then were rescued under DAPA treatment (Figure 4(e)), supporting the autophagy pathway activation under DAPA stimulation in vitro. Moreover, western blotting illustrated the upregulation of p-AMPK protein abundance and downregulation of p-mTOR protein abundance in H9C2 cells under hypoxia relative to controls and were reversed after DAPA treatment (Figure 4(f)). Collectively, DAPA suppresses hypoxia-treated H9C2 cell apoptosis in vitro through autophagy activation.

### 3.5. DAPA Represses Hypoxia-Induced H9C2 Cell Apoptosis via the AMPK/mTOR Pathway

To validate the AMPK/mTOR influence on the H9C2 cell apoptosis, we conducted rescue assays using Comp C, an inhibitor of AMPK. We discovered that the decreased apoptosis rate of hypoxia-treated H9C2 cells under DAPA was rescued by Comp C (Figure 5(a)). There was a similar trend of the caspase-3/7 expression through western blotting and caspase-3 expression through IF staining (Figures 5(b) and 5(c)). Collectively, DAPA suppresses hypoxia-treated H9C2 cell apoptosis via the AMPK/mTOR pathway.

RETRACTED

## 4. Discussion

VR refers to the molecular, cellular, and interstitial changes caused by myocardial injury or cardiac pressure load, resulting in changes in cardiac wall thickness, ventricular volume, and cardiac mass [22]. Lee et al. dilated using a balloon dilatation catheter and injured the abdominal aorta of nondiabetic New Zealand white rabbits fed with high cholesterol diet and then intervened the rabbits with DAPA or placebo for 8 weeks; they discovered that dapagliflozin can suppress inflammation and macrophage activity to exert an antiatherosclerotic role [23]. More importantly, it has been reported that DAPA can reduce the risk of worsening HF [15]. Nevertheless, there are few reports on DAPA on VR. VR involves changes in cardiac geometry and function, manifested by decreased LVEF and increased left ventricular volume or mass [24]. Changes in heart size and shape can predict the prognosis of HF and assess response to therapy [25, 26]. Herein, ligation of LAD-triggered HF was used to establish nondiabetic rat HF models, and its pathophysiological changes were similar to those of hypoxic HF patients. We discovered that model rats presented unarranged left ventricular myocardial fibers and unordered cell morphology, while DAPA rescued these pathological changes. Additionally, model rats presented elevation in HW, LVW, HW/TL, and LVW/TL as well as plasma ANP and BNP levels while DAPA rescued these changes. Furthermore, DAPA also reversed the structural changes and systolic and diastolic dysfunction in model rats. These finding suggested that DAPA hinders left VR and benefits cardiac function in HF progression, which was in line with the study proposed by Zhang et al. They have demonstrated that DAPA improves left VR and aorta sympathetic tone in a pig model of HF [27].

Autophagy exerts a crucial role in maintaining cardiac homeostasis and function [28]. In recent years, autophagy has revealed to have relation to occurrence and development of HF [29]. Beclin-1 and LC3II protein levels in heart tissue of chronic HF patients presented elevation, and both of them presented downregulation after application of left ventricular assist device [30]; in HF mice induced by adriamycin, a large number of autophagosome structures were observed [31]; Nakai et al. specifically knocked down autophagy gene ATG5 in mice, and then cardiac function of mice presented depletion [32]. These reports suggest that autophagy has close association with HF. Herein, LC3B-II/I and beclin-1 protein abundances presented depletion, whereas p62 showed upregulation in myocardial tissue of model rats and then were rescued under DAPA treatment. LC3B-II/I and beclin-1 protein abundances presented depletion, whereas p62 showed upregulation in H9C2 cells under hypoxia and then were rescued under DAPA treatment. These findings suggested that DAPA exerts a promoting influence on autophagy in HF. In HF, autophagy activation can specifically remove reactive oxygen species and inflammatory cytokines and reduce myocardial cell apoptosis [33], preventing further deterioration of cardiac function. Herein, cardiomyocyte apoptosis rate and caspase-3/7 levels in myocardial tissue of model rats presented elevation, whereas DAPA treatment reversed this effect. Hypoxia triggered the elevation of H9C2 cell apoptosis and DAPA countervailed this influence. These findings suggested that DAPA exerts an inhibitory influence on cardiomyocyte apoptosis in HF through activating autophagy. Consistent with our results, previous studies have also indicated the alleviating role of DAPA in many diseases through activating autophagy. For instance, DAPA activates autophagy to attenuate inflammatory bowel disease in rats [34]. DAPA improves pancreatic injury and promotes kidney autophagy via the AMPK/mTOR signaling pathway [35]. It has been revealed that AMPK phosphorylates and activates ULK1, triggering the initiation of autophagic cascade [36, 37]. Importantly, mTOR strongly suppresses autophagy through direct phosphorylation and ULKI inhibition [38]; thus, AMPK facilitates autophagy not only by directly activating ULK1 but also by negatively regulating mTORCI and blocking its inhibitory effect on ULKI. Additionally, activation of AMPK/mTOR-mediated autophagy can also reduce collagen deposition and reduce myocardial fibrosis [39]. Moreover, DAPA has been proved to alleviate hepatic steatosis by the AMPK/mTOR pathway [17]. Yang et al. have pointed that DAPA reduces advanced glycation end product triggered podocyte injury by the AMPK/mTOR pathway [40]. Herein, p-AMPK protein presented downregulation and of p-mTOR protein presented upregulation in myocardial tissue of model rats and were reversed after DAPA treatment. p-AMPK protein presented upregulation and of p-mTOR protein presented downregulation in H9C2 cells under hypoxia and were reversed after DAPA treatment. Moreover, Comp C, a cell-permeable pyrazole derivative, is widely used as an inhibitor of AMPK to characterize the role of AMPK in physiological processes [41]. Our rescue assays demonstrated that the decreased apoptosis rate and caspase-3/7 expression in hypoxia-treated H9C2 cells under DAPA was rescued by Comp C. Thus, DAPA-induced autophagy activation can reduce cardiomyocyte apoptosis via the AMPK/mTOR pathway, thereby delaying HF progression.

RETRACTED

There are some limitations in our study. First, our results suggest that DAPA activated the AMPK/mTOR pathway, but it is not clear how this step is completed. In addition, we cannot rule out the effects of other mechanisms that DAPA improves HF in addition to the mechanisms examined here. Therefore, further research is essential to examine the above limitations in more depth.

In conclusion, DAPA suppresses ventricular remodeling in HF through activating autophagy via AMPK/mTOR pathway, providing a potential novel insight for seeking therapeutic plans of HF.

## Figures and Tables

**Figure 1:** DAPA attenuated left VR and improved cardiac function in HF rats. (a) HE staining assessed histopathological changes in left ventricular myocardial tissue of rats in control, model, or DAPA group. (b), Quantitative analysis of cardiomyocyte diameter in left ventricular tissue of rats in each group. (c)–(f) Quantitative analysis of HW, LVW, HW/TL ,and LVW/TL of rats in each group. (g, h) ELISA measured plasma ANP and BNP levels of rats in each group. (i) M-mode echocardiography detected cardiac function of rats in each group. (j)–(m) Quantitative analysis of LVIDs, LVIDd, EF, and FS of rats in each group. ^∗∗^*p* < 0.01, ^∗∗∗^*p* < 0.001; ^#^*p* < 0.05, ^##^*p* < 0.01.

**Figure 2:** DAPA attenuated cardiomyocyte apoptosis in HF rats. (a) Apoptosis of infarct margin cells in myocardial tissue of rats in control, model, or DAPA group. Data are derived from TUNEL staining assay. (b) Western blot detected levels of apoptosis-related proteins in myocardial tissue of rats in each group. (c) Caspase-3 level in myocardial tissue of rats in each group. Data are derived from immunohistochemical staining assay. ^∗∗^*p* < 0.01, ^∗∗∗^*p* < 0.001; ^#^*p* < 0.05, ^##^*p* < 0.01, ^###^*p* < 0.001.

**Figure 3:** DAPA facilitated cardiomyocyte autophagy in HF rats via the AMPK/mTOR pathway. (a) Immunohistochemical staining detected LC3B level in myocardial tissue of rats in control, model, or DAPA group. (b) Western blot detected levels of autophagy-related proteins in myocardial tissue of rats in each group. (c) Western blot detected levels of AMPK/mTOR-related proteins in myocardial tissue of rats in each group. ^∗∗∗^*p* < 0.001; ^##^*p* < 0.01, ^###^*p* < 0.001.

**Figure 4:** DAPA repressed hypoxia-induced H9C2 cell apoptosis by facilitating autophagy. (a) Flow cytometry detected H9C2 cell apoptosis in control, H/R, or H/R + DAPA group. (b) Western blot detected levels of apoptosis-related proteins in H9C2 cells under different conditions. (c) Immunofluorescence detected caspase-3 level in H9C2 cells under different conditions. (d) Immunofluorescence detected LC3B level in H9C2 cells under different conditions. (e) Western blot detected levels of autophagy-related proteins in H9C2 cells under different conditions. (f) Western blot detected levels of AMPK/mTOR-related proteins in H9C2 cells under different conditions. ^∗∗∗^*p* < 0.001; ^#^*p* < 0.05, ^##^*p* < 0.01, ^###^*p* < 0.001.

RETRACTED

**Figure 5:** DAPA repressed hypoxia-induced H9C2 cell apoptosis via the AMPK/mTOR pathway. (a) Flow cytometry detected H9C2 cell apoptosis in control, H/R, H/R + DAPA, or H/R + DAPA+Comp C group. (b) Western blot detected levels of apoptosis-related proteins in H9C2 cells under different conditions. (c) Immunofluorescence detected caspase-3 level in H9C2 cells under different conditions. ^∗∗∗^*p* < 0.001; ^###^*p* < 0.001; ^&&^*p* < 0.01, ^&&&^*p* < 0.001.

## Data Availability

Data generated in this study are available from the corresponding author under reasonable request.
